# A Novel Multistep Iterative Technique for Models in Medical Sciences with Complex Dynamics

**DOI:** 10.1155/2022/7656451

**Published:** 2022-07-28

**Authors:** Sania Qureshi, Amanullah Soomro, Asif Ali Shaikh, Evren Hincal, Nezihal Gokbulut

**Affiliations:** ^1^Mehran University of Engineering and Technology, Department of Basic Sciences and Related Studies, Jamshoro 76062, Pakistan; ^2^Near East University, Department of Mathematics, Mersin 10, Turkey; ^3^Near East University, Mathematics Research Center, Mersin 10, Turkey

## Abstract

This paper proposes a three-step iterative technique for solving nonlinear equations from medical science. We designed the proposed technique by blending the well-known Newton's method with an existing two-step technique. The method needs only five evaluations per iteration: three for the given function and two for its first derivatives. As a result, the novel approach converges faster than many existing techniques. We investigated several models of applied medical science in both scalar and vector versions, including population growth, blood rheology, and neurophysiology. Finally, some complex-valued polynomials are shown as polynomiographs to visualize the convergence zones.

## 1. Introduction

Numerical analysis is an area of computer science and mathematics that implements, analyses, and develops methods for solving numerical problems in applied mathematics. Researchers have devised many iterative techniques for solving nonlinear equations of the kind *ζ*(*x*) = 0, used as models in medical science areas like blood rheology, non-Newtonian mechanics, fluid dynamics, population dynamics, and neurophysiology. Many researchers have found that methods can be combined to design modified iterative techniques for solving nonlinear problems in a wide range of fields, including engineering and science. Some of the recent works can be found in [1–11] and the references cited therein.

We developed and examined some iterative techniques for solving nonlinear equations in the field of applied medical science. The convergence order, number of iterations, number of function evaluations, and the precision of the desired root are the most important factors to consider when determining or measuring the performance of an iterative method. Because each iterative method works differently for each nonlinear equation. A method that costs the least time and still has the best root accuracy is the most efficient.

This study was aimed at establishing a novel hybrid three-step iterative technique for solving both scalar and vector form of nonlinear equations that arise in several fields of science and engineering. In addition to several existing techniques, we attempted to establish a new three-step numerical technique by blending a third-order method [12, 13] with the standard second-order Newton-Raphson method. This blending resulted in a sixth-order technique requiring only five functional evaluations per iterations—three functions *ζ*(*x*) = 0 and two for its first-order derivatives *ζ*′(*x*) = 0. It may be noted that the major motivation lying behind the development of the proposed three-step method is the accelerated sixth-order of convergence while maintaining the computational cost. With the proposed method, one can handle the numerical problems that arise in [14–18] and the similar works.

This paper is structured as follows: Section 2 explains the computational complexity and steps for some existing methods.  Section 3 describes the formulation of the proposed three-step iterative technique.  Section 4 explains the convergence order for the technique in both scalar and vector forms of the function.  Section 5 has details on the polynomiography. Some numerical tests containing applied medical science models are presented in Section 6. Finally, the research work is concluded with a few research directions that are given in Section 7.

## 2. Existing Iterative Methods

The Newton-Raphson approach *N*2 in [13] has a quadratic order of convergence. This existing approach is the most commonly used root-finding approach among several existing ones. Its computational process is represented below, and it involves two function evaluations: one for the function itself and another for the first-order derivative of the function

(1) $$\begin{array}{c} x_{n+1}=x_{n}-\frac{\zeta \left(x_{n}\right)}{\zeta^{\prime }\left(x_{n}\right)},n=0,1,2,\cdots , \end{array}$$

where *ζ*′(*x*_*n*_) ≠ 0. In [19], researchers developed a modified version of an existing approach aimed at reducing first-order derivatives. They devised a two-step approach with fourth-order convergence, denoted as *N*4. One of the algorithm's advantages was the usage of only four function evaluations per iteration, as seen in the computational structure below:

(2) $$\begin{array}{c} y_{n}=x_{n}-\frac{\zeta \left(x_{n}\right)}{\sigma \left(x_{n}\right)},\\ x_{n+1}=y_{n}-\frac{\zeta \left(y_{n}\right)}{\sigma \left(y_{n}\right)}-\frac{\zeta^{2}\left(y_{n}\right)\zeta \left(x_{n},y_{n}\right)}{2\zeta^{3}\left(y_{n}\right)},\\ n=0,1,\cdots , \end{array}$$

where

(3) $$\begin{array}{c} \sigma \left(x_{n}\right)=\frac{\zeta \left(x_{n}+\zeta \left(x_{n}\right)\right)-\zeta \left(x_{n}\right)}{\zeta \left(x_{n}\right)},\\ \sigma \left(y_{n}\right)=\frac{\zeta \left(y_{n}+\zeta \left(y_{n}\right)\right)-\zeta \left(y_{n}\right)}{\zeta \left(y_{n}\right)},\\ \zeta \left(x_{n},y_{n}\right)=\frac{\sigma \left(y_{n}\right)-\sigma \left(x_{n}\right)}{\zeta \left(y_{n}\right)-\zeta \left(x_{n}\right)}. \end{array}$$

The use of a three-step iterative method to get sixth-order convergence is suggested in this study.

The authors in [20] have blended two different approaches. Their method combines the second- and third-order approach described in the reference. Three function evaluations are required at the start of the procedure, followed by two first-order derivative evaluations for each iteration after that. The notation *N*6 is used to denote this method, and the computational steps to represent the method are as follows:

(4) $$\begin{array}{c} y_{n}=x_{n}-\frac{\zeta \left(x_{n}\right)}{\zeta^{\prime }\left(x_{n}\right)},\\ z_{n}=y_{n}-\frac{\zeta \left(y_{n}\right)}{\zeta^{\prime }\left(y_{n}\right)},\\ x_{n+1}=y_{n}-\frac{\zeta \left(y_{n}\right)+\zeta \left(z_{n}\right)}{\zeta^{\prime }\left(y_{n}\right)},\\ n=0,1,2,\cdots . \end{array}$$

In [21], the authors proposed two three-step approaches with the same order of convergence. Both approaches have sixth-order, requiring three function evaluations and two first-order derivatives per iteration. Both approaches are described in the following equations:

(5) $$\begin{array}{c} y_{n}=x_{n}-\frac{\zeta \left(x_{n}\right)}{\zeta^{\prime }\left(x_{n}\right)}, \end{array}$$

(6) $$\begin{array}{c} z_{n}=y_{n}-\frac{\zeta \left(y_{n}\right)}{\zeta^{\prime }\left(y_{n}\right)}, \end{array}$$

## 3. Proposed Iterative Technique

In this section, the objective is to introduce a modified iterative method while using the idea of amalgamation of two existing methods having convergence orders *ρ*_1_ and *ρ*_2_. The concept of mixing two existing iterative methods to yield a method with better accuracy having order *ρ*_1_*ρ*_2_ has been employed in number of research works conducted in recent past, including [4, 5, 20, 22] and some of the references cited therein. Being motivated with such studies, we attempt here to blend the most frequently used Newton-Raphson method having second-order convergence with a third-order method given in [23] to obtain an iterative method of sixth-order convergence as shown below:

(7) $$\begin{array}{c} y_{n}=x_{n}-\frac{\zeta \left(x_{n}\right)}{\zeta^{\prime }\left(x_{n}\right)},\\ z_{n}=y_{n}-\frac{\zeta \left(y_{n}\right)}{\zeta^{\prime }\left(y_{n}\right)},\\ x_{n+1}=z_{n}-\left(1+2{\left(\frac{\zeta \left(y_{n}\right)}{\zeta \left(x_{n}\right)}\right)}^{2}+\frac{2\zeta \left(z_{n}\right)}{\zeta \left(y_{n}\right)}\right)\frac{\zeta \left(z_{n}\right)}{\zeta^{\prime }\left(y_{n}\right)},\\ \;n=0,1,2,\cdots . \end{array}$$

The flowchart of the above sixth-order proposed three-step iterative method is shown in Figure 1.

## 4. Order of Convergence

This section is dedicated to the theoretical proof for the order of convergence of the proposed three-step iterative method (7) in both scalar and vector forms. The well-known Taylor series for a function of single and multivariable will be used to achieve the required results.

### 4.1. Convergence Theory with Scalar Form

In this subsection, we theoretically prove the local order of convergence for the scalar form of a nonlinear equation, that is, *ζ*(*x*) = 0, for the proposed three-step sixth-order method given in (7).

**Theorem 1 .**

Suppose that *γ* ∈ *P* is the exact root of a differentiable function *ζ* : *P* ⊂ ℝ⟶ℝ for an open interval *P*. Then, the three-step proposed method given in (7) has sixth-order convergence, and the asymptotic error term is determined to be

(8) $$\begin{array}{c} e_{n+1}=-\frac{2d_{2}^{5}}{d_{1}^{5}}e_{n}^{6}+O\left(e_{n}^{7}\right), \end{array}$$

where *e*_*n*_ = *x*_*n*_ − *γ*, and *d*_*r*_ = *ζ*^*r*^(*γ*)/*r*!, *r* = 1, 2, 3, ⋯.

**Proof**

Suppose that *γ* is the exact root of the function *ζ*(*x*_*n*_), where *x*_*n*_ is the approximate term at the *n*th iteration to the root by the proposed method of order six and *e*_*n*_ = *x*_*n*_ − *γ* is the error term after the *n*th iteration. Applying Taylor series for function *ζ*(*x*_*n*_) about *γ*, we have obtained the following expansion:

(9) $$\begin{array}{c} \zeta \left(x_{n}\right)=d_{1}e_{n}+d_{2}e_{n}^{2}+O\left(e_{n}^{3}\right). \end{array}$$

Applying Taylor series for function 1/(*ζ*′(*x*_*n*_)) about *γ*, we have

(10) $$\begin{array}{c} \frac{1}{\zeta^{\prime }\left(x_{n}\right)}=\frac{-3d_{1}d_{3}e_{n}^{2}+4d_{2}^{2}e_{n}^{2}-2d_{1}d_{2}e_{n}+d_{1}^{2}}{d_{1}^{3}}+O\left(e_{n}^{3}\right). \end{array}$$

Multiplying (9) and (10), we obtain

(11) $$\begin{array}{c} \frac{\zeta \left(x_{n}\right)}{\zeta^{\prime }\left(x_{n}\right)}=\frac{e_{n}\left(d_{2}e_{n}+d_{1}\right)\left(-3d_{1}d_{3}e_{n}^{2}+4d_{2}^{2}e_{n}^{2}-2d_{1}d_{2}e_{n}+d_{1}^{2}\right)}{d_{1}^{3}}. \end{array}$$

Substituting (11) in the first step of (7), we obtain

(12) $$\begin{array}{c} \hat{e_{n}}=\frac{e_{n}^{2}\left(3d_{1}d_{2}d_{3}e_{n}^{2}-4d_{2}^{3}e_{n}^{2}+3d_{1}^{2}d_{3}e_{n}-2d_{1}d_{2}^{2}e_{n}+d_{2}d_{1}^{2}\right)}{d_{1}^{3}}, \end{array}$$

where $\hat{e_{n}}=y_{n}-\gamma$. Using the Taylor's series for *ζ*(*y*_*n*_) around *γ*, we obtain

(13) $$\begin{array}{c} \zeta \left(y_{n}\right)=d_{1}\hat{e_{n}}+d_{2}{\overset{\wedge }{e_{n}}}^{2}+O\left({\overset{\wedge }{e_{n}}}^{3}\right). \end{array}$$

Applying Taylor series for the function 1/(*ζ*′(*y*_*n*_)) about *γ*, we have

(14) $$\begin{array}{c} \frac{1}{\zeta^{\prime }\left(y_{n}\right)}=\frac{-3d_{1}d_{2}{\overset{\wedge }{e_{n}}}^{2}+4d_{2}^{2}{\overset{\wedge }{e_{n}}}^{2}-2d_{1}d_{1}\hat{e_{n}}+d_{1}^{2}}{d_{1}^{3}}+O\left({\overset{\wedge }{e_{n}}}^{3}\right). \end{array}$$

Multiplying (13) and (14), we obtain

(15) $$\begin{array}{c} \frac{\zeta \left(y_{n}\right)}{\zeta^{\prime }\left(y_{n}\right)}=\frac{\hat{e_{n}}\left(d_{2}\hat{e_{n}}+d_{1}\right)\left(-3d_{1}d_{3}{\overset{\wedge }{e_{n}}}^{2}+4d_{2}{\overset{\wedge }{e_{n}}}^{2}-2d_{1}d_{2}\hat{e_{n}}+d_{1}^{2}\right)}{d_{1}^{3}}. \end{array}$$

Substituting (15) in the second step of (7), we obtain

(16) $$\begin{array}{c} \tilde{e_{n}}=\frac{{\overset{\wedge }{e_{n}}}^{2}\left(3d_{1}d_{2}d_{3}{\overset{\wedge }{e_{n}}}^{2}-4d_{2}^{3}{\overset{\wedge }{e_{n}}}^{2}+3d_{1}^{2}d_{3}\hat{e_{n}}-2d_{1}d_{2}^{2}\hat{e_{n}}+d_{2}d_{1}^{2}\right)}{d_{1}^{3}}, \end{array}$$

where $\tilde{e_{n}}=z_{n}-\gamma$. Using the Taylor's series *ζ*(*z*_*n*_) around *γ*, we obtain

(17) $$\begin{array}{c} \zeta \left(z_{n}\right)=d_{1}\tilde{e_{n}}+d_{2}{\tilde{e_{n}}}^{2}+O\left({\tilde{e_{n}}}^{3}\right). \end{array}$$

Applying Taylor series for function 1/(*ζ*(*x*_*n*_)) about *γ*, we have

(18) $$\begin{array}{c} \frac{1}{\zeta \left(x_{n}\right)}=\frac{d_{2}^{2}e_{n}^{2}-d_{1}d_{2}e_{n}+d_{1}^{2}}{d_{1}^{3}e_{n}}. \end{array}$$

Applying Taylor series for function 1/(*ζ*(*y*_*n*_)) about *γ*, we have

(19) $$\begin{array}{c} \frac{1}{\zeta \left(y_{n}\right)}=\frac{d_{2}^{2}{\overset{\wedge }{e_{n}}}^{2}-d_{1}d_{2}\hat{e_{n}}+d_{1}^{2}}{d_{1}^{3}\hat{e_{n}}}. \end{array}$$

Substituting (13), (14), (17), (18), and (19) in the third step of (7), one obtains

(20) $$\begin{array}{c} e_{n+1}=\frac{\left(-2{\overset{\wedge }{e_{n}}}^{2}\tilde{e_{n}}{\left(d_{2}\overset{\wedge }{e_{n}}+d_{1}\right)}^{2}\left(d_{2}\hat{e_{n}}+d_{1}\right)\left(-3d_{1}d_{3}{\overset{\wedge }{e_{n}}}^{2}+4d_{2}^{2}{\overset{\wedge }{e_{n}}}^{2}-2d_{1}d_{2}\hat{e_{n}}+d_{1}^{2}\right)\left(-2d_{2}e_{n}+d_{1}\right)\right)}{d_{1}^{6}e_{n}^{2}}. \end{array}$$

Finally, using Equations (12) and (16), we obtain the required results as follows:

(21) $$\begin{array}{c} e_{n+1}=-\frac{2d_{2}^{5}}{d_{1}^{5}}e_{n}^{6}+O\left(e_{n}^{7}\right). \end{array}$$

Hence, the sixth-order convergence of the proposed three-step iterative method given by (7) for the nonlinear functions in single variable (*ζ*(*x*) = 0) is proved.

### 4.2. Convergence Theory with Vector Form

In this subsection, we theoretically prove the local order of convergence for the vector form of a nonlinear equation, that is, *ζ*(*x*) = 0, where *ζ* : *P* ⊂ ℝ^*N*^⟶ℝ^*N*^ is a sufficiently Frechet differentiable function and *N* shows the number of unknowns in the system of nonlinear equations. The proposed three-step method given in (7) is shown below in its vector version:

(22) $$\begin{array}{c} y_{n}=x_{n}-\zeta^{\prime }{\left(x_{n}\right)}^{-1}\zeta \left(x_{n}\right),\\ z_{n}=y_{n}-\zeta^{\prime }{\left(y_{n}\right)}^{-1}\zeta \left(y_{n}\right),\\ x_{n+1}=z_{n}-\left(1+2{\left(\zeta^{\prime }{\left(x_{n}\right)}^{-1}\zeta \left(y_{n}\right)\right)}^{2}+2\left(\zeta {\left(y_{n}\right)}^{-1}\zeta \left(z_{n}\right)\right)\left(\zeta {\left(y_{n}\right)}^{-1}\zeta \left(z_{n}\right)\right)\right), \end{array}$$

where *ζ*′ stands for the Jacobian matrix of *ζ*.

**Lemma 1 .**

Let *ζ* : *Π* ⊂ ℝ^*N*^⟶ℝ^*N*^ be an *r*-times Frechet differentiable in a convex set *Π* ⊂ ℝ^*N*^. Then, for any *x* and *h* ∈ ℝ^*N*^, the following expression holds.

(23) $$\begin{array}{c} \zeta \left(x+h\right)=\zeta \left(x\right)+\zeta^{\prime }\left(x\right)h+\frac{1}{2!}\zeta^{\prime \prime }\left(x\right)h^{2}+\frac{1}{3!}\zeta^{\prime \prime }\left(x\right)h^{3}+\cdots +\frac{1}{r!}\zeta^{\left(r-1\right)}\left(x\right)h^{r-1}+R_{r}, \end{array}$$

where $\left\|R_{r}\right\|\leq \underset{0<t<1}{\sup}\left\|\zeta^{\left(r\right)}\left(x+ht\right)\right\|{\left\|h\right\|}^{r}$.

We present the following theorem to show the error equation and thus the order of convergence for the proposed three-step method given in (7) in case of a system of nonlinear equations (vector form).

**Theorem 2 .**

Let the function *ζ* : *Π* ⊂ ℝ^*N*^⟶ℝ^*N*^ be sufficiently differentiable in a convex set *Π* containing a simple zero $\overset{⟶}{\gamma }$ of *ζ*(*x*). Let us consider that *ζ*′(*x*) is continuous and nonsingular in $\overset{⟶}{\gamma }$. If the initial guess *x*_0_ is close to $\overset{⟶}{\gamma }$, then the sequence {*x*_*n*_} obtained with the proposed three-step method given in (7) converges to $\overset{⟶}{\gamma }$ with sixth-order of convergence.

**Proof**

Suppose that $\overset{⟶}{\gamma }$ is the exact root of the function *ζ*(*x*_*n*_), *x*_*n*_ is the *n*th term approximation to the exact root by proposed method, and $e_{n}=x_{n}-\overset{⟶}{\gamma }$ is the error term after the *n*th iteration, and $D_{r}=\zeta^{\left(r\right)}\left(\overset{⟶}{\gamma }\right)/r!,r=1,2,3,\cdots$.

Applying Taylor series for the vector function *ζ*(*x*_*n*_) about $\overset{⟶}{\gamma }$, we have obtained the following:

(24) $$\begin{array}{c} \zeta \left(x_{n}\right)=D_{1}e_{n}+D_{2}e_{n}^{2}+O\left(e_{n}^{3}\right). \end{array}$$

Applying Taylor series for the inverted Jacobian matrix *ζ*′(*x*_*n*_)^−1^ about $\overset{⟶}{\gamma }$, we have

(25) $$\begin{array}{c} \zeta^{\prime }{\left(x_{n}\right)}^{-1}=\frac{-3D_{1}D_{3}e_{n}^{2}+4D_{2}^{2}e_{n}^{2}-2D_{1}D_{2}e_{n}+D_{1}^{2}}{D_{1}^{3}}+O\left(e_{n}^{3}\right). \end{array}$$

Multiplying (24) and (25), we obtain

(26) $$\begin{array}{c} \zeta^{\prime }{\left(x_{n}\right)}^{-1}\zeta \left(x_{n}\right)=\frac{e_{n}\left(D_{2}e_{n}+D_{1}\right)\left(-3D_{1}D_{3}e_{n}^{2}+4D_{2}^{2}e_{n}^{2}-2D_{1}D_{2}e_{n}+D_{1}^{2}\right)}{D_{1}^{3}}. \end{array}$$

Substituting (26) in the first step of (7), we obtain

(27) $$\begin{array}{c} \hat{e_{n}}=\frac{e_{n}^{2}\left(3D_{1}D_{2}D_{3}e_{n}^{2}-4D_{2}^{3}e_{n}^{2}+3D_{1}^{2}D_{3}e_{n}-2D_{1}D_{2}^{2}e_{n}+D_{2}D_{1}^{2}\right)}{D_{1}^{3}}, \end{array}$$

where $\hat{e_{n}}=y_{n}-\overset{⟶}{\gamma }$. Using the Taylor's series for *ζ*(*y*_*n*_) around $\overset{⟶}{\gamma }$, we obtain

(28) $$\begin{array}{c} \zeta \left(y_{n}\right)=D_{1}\hat{e_{n}}+D_{2}{\overset{\wedge }{e_{n}}}^{2}+O\left({\overset{\wedge }{e_{n}}}^{3}\right). \end{array}$$

Applying Taylor series for function *ζ*′(*y*_*n*_)^−1^ about $\overset{⟶}{\gamma }$, we have

(29) $$\begin{array}{c} \zeta^{\prime }{\left(y_{n}\right)}^{-1}=\frac{-3D_{1}D_{3}{\overset{\wedge }{e_{n}}}^{2}+4D_{2}^{2}{\overset{\wedge }{e_{n}}}^{2}-2D_{1}D_{2}\hat{e_{n}}+D_{1}^{2}}{D_{1}^{3}}+O\left({\overset{\wedge }{e_{n}}}^{3}\right). \end{array}$$

Multiplying (28) and (29), we obtain

(30) $$\begin{array}{c} \zeta^{\prime }{\left(y_{n}\right)}^{-1}\zeta \left(y_{n}\right)=\frac{\hat{e_{n}}\left(D_{2}\hat{e_{n}}+D_{1}\right)\left(-3D_{1}D_{3}{\overset{\wedge }{e_{n}}}^{2}+4D_{2}^{2}{\overset{\wedge }{e_{n}}}^{2}-2D_{1}D_{2}\hat{e_{n}}+D_{1}^{2}\right)}{D_{1}^{3}}. \end{array}$$

Substituting (30) in the second step of (7), we obtain

(31) $$\begin{array}{c} \tilde{e_{n}}=\frac{{\overset{\wedge }{e_{n}}}^{2}\left(3D_{1}D_{2}D_{3}{\overset{\wedge }{e_{n}}}^{2}-4D_{2}^{3}{\overset{\wedge }{e_{n}}}^{2}+3D_{1}^{2}D_{3}\hat{e_{n}}-2D_{1}D_{2}^{2}\hat{e_{n}}+D_{2}D_{1}^{2}\right)}{D_{1}^{3}}, \end{array}$$

where $\tilde{e_{n}}=z_{n}-\overset{⟶}{\gamma }$. Using the Taylor's series for *ζ*(*z*_*n*_) around $\overset{⟶}{\gamma }$, we obtain

(32) $$\begin{array}{c} \zeta \left(z_{n}\right)=D_{1}\tilde{e_{n}}+D_{2}{\tilde{e_{n}}}^{2}+O\left({\tilde{e_{n}}}^{3}\right). \end{array}$$

Applying Taylor series for function *ζ*(*x*_*n*_)^−1^ about $\overset{⟶}{\gamma }$, we have

(33) $$\begin{array}{c} \zeta {\left(x_{n}\right)}^{-1}=\frac{D_{2}e_{n}^{2}-D_{2}e_{n}D_{1}+D_{1}^{2}}{D_{1}^{3}e_{n}}. \end{array}$$

Applying Taylor series for function *ζ*(*y*_*n*_)^−1^ about $\overset{⟶}{\gamma }$, we have

(34) $$\begin{array}{c} \zeta {\left(y_{n}\right)}^{-1}=\frac{D_{2}{\overset{\wedge }{e_{n}}}^{2}-D_{2}\hat{e_{n}}D_{1}+D_{1}^{2}}{D_{1}^{3}\hat{e_{n}}}. \end{array}$$

Substituting (14), (28), (32), (33), and (34) in the third step of the proposed method (7), one obtains

(35) $$\begin{array}{c} e_{n+1}=\frac{\left(-2{\overset{\wedge }{e_{n}}}^{2}\tilde{e_{n}}{\left(D_{2}\overset{\wedge }{e_{n}}+D_{1}\right)}^{2}\left(D_{2}\hat{e_{n}}+D_{1}\right)\left(-3D_{1}D_{3}{\overset{\wedge }{e_{n}}}^{2}+4D_{2}^{2}{\overset{\wedge }{e_{n}}}^{2}-2D_{1}D_{2}\hat{e_{n}}+D_{1}^{2}\right)\left(-2D_{2}e_{n}+D_{1}\right)\right)}{D_{1}^{6}e_{n}^{2}}. \end{array}$$

Using (27) and (31) in the above equation, we obtain

(36) $$\begin{array}{c} e_{n+1}=-\frac{2D_{2}^{5}}{D_{1}^{5}}e_{n}^{6}+O\left(e_{n}^{7}\right). \end{array}$$

Hence, the sixth-order convergence of the proposed three-step iterative method given by (7) for the nonlinear functions in multivariable case (*ζ*(*x*) = 0) is proved.

## 5. Polynomiography with Proposed Technique

Polynomiography is incredibly useful in arts, education, and applied medical science, visualizing complicated polynomial zeros through the use of fractal and nonfractal images generated by iterative processes on a two-dimensional plane. An individualized image is known as “polynomiograph.” At the beginning of the 20th century, Dr. Bahman Kalantari introduced the term “polynomiography.” His research on polynomial root-finding, an old traditional field that continues to yield new insights with each successive generation of academics, mathematicians, and physicists, inspired the concepts for polynomiography. It is an iterative process for making two-dimensional colored images (polynomiographs) that show behavior of initial estimates towards the roots of polynomials.

We employ a rectangle *ℛ* ∈ *ℂ* over a meshgrid [−1.5, 1.5] × [−1.5, 1.5] with tolerance (*ϵ* = 10^−3^) and the maximum number of iterations are taken as *N* = 20 to generate polynomiographs over the complex plane *ℂ*. With the help of several available software such as Python, MATLAB, and Mathematica, it is possible to generate polynomiographs over the complex plane *ℂ* of different complex-valued polynomials. The different colors can be assigned to roots, while the convergence can be observed with the change in assigned colors. The way we divide the meshgrid affects the pixel density of the visual representations we make. For example, if we divide *ℛ* into a grid of 5000 × 5000, the plotted polynomiographs will have outstanding resolution, and this is what has been done for the following complex-valued polynomials in Figure 2.

(37) $$\begin{array}{c} \left(a\right)\;Q_{1}\left(z\right)=z^{3}-1,\\ \left(b\right)\;Q_{2}\left(z\right)=z^{4}-1,\\ \left(c\right)\;Q_{3}\left(z\right)=35z^{9}-180z^{7}+378z^{5}-420z^{3}+315z,\\ \left(d\right)\;Q_{4}\left(z\right)=z^{10}-1. \end{array}$$

## 6. Medical Science Models for Numerical Simulations

This section carries out numerical simulations for some important and frequently used models in the fields of medical science. These models are represented as nonlinear equations in single and several unknowns so that one can find the approximate solutions. It may be noted that the exact solution may not be possible to find due to the nonlinearity, and we have to go for iterative methods as mentioned before. The iterative methods under consideration are listed in the Section 2. Thus, we have six iterative techniques, the proposed inclusive. For the purpose of simulations and comparison, the tolerance is set as *ϵ* = 10^−300^ as a stopping criterion with 12000 digits of precision, while different numbers of iterations are used with varying values of the initial guesses under MAPLE software.

**Problem 1 (blood rheology model [24]).**

The physical and flow characteristics of the blood are studied in the area of medical science called the blood rheology. Blood, being a Non-Newtonian fluid, is considered as a Caisson fluid whose model demonstrates that the flow in a tube moves as a plug with little deformation and velocity gradient occurs near the wall. To investigate the plug flow of Caisson fluid flow, we consider the following nonlinear equation:

(38) $$\begin{array}{c} \zeta_{1}\left(x\right)=\frac{x^{8}}{441}-\frac{8x^{5}}{63}-0.05714285714x^{4}+\frac{16x^{2}}{9}-3.624489796x+0.36, \end{array}$$

where *x* shows the plug flow of Caisson fluid flow.

It is observed in Table 1 that the absolute error at the final iteration is smallest of all the errors and so is the absolute functional value while consuming reasonable amount of machine time computed in seconds. It is true in case of both initial guesses, that is, *x*_0_ = 2.0 and *x*_0_ = 4.2. For the first initial guess, the number of iterations is set to *N* = 6, and it is *N* = 5 for the second initial guess. However, the absolute errors are smallest for the proposed method in both situations. Further, it may also be noted that the method given in Equation (5) diverges for *x*_0_ = 2.0, while it converges for the second initial guess. Similarly, the method given in Equation (2) converges to the solution other than the required one.

**Problem 2 (law of blood flow [25]).**

This law is given by French physician Jean Louis-Marie Poiseuille in 1840. The blood flows through the vein or artery, where *η* is the viscosity of blood, *R* is the radius, *l* is the length, *P* is the pressure, and *ζ* is the function of *x* with the domain [0, *R*]. This law, when stated, turns into the following nonlinear model:

(39) $$\begin{array}{c} \zeta_{2}\left(x\right)=\frac{P}{\eta l}\left(R^{2}-x^{2}\right), \end{array}$$

where *P* = 4000, *η* = 0.027, *R* = 0.008, and *l* = 2 are chosen for the simulations with *x* ∈ [0, *R*] being the distance to be determined.

It is observed in Table 2 that the absolute error at the final iteration is smallest of all the errors and so is the absolute functional value while consuming reasonable amount of machine time computed in seconds. It is true in case of both initial guesses, that is, *x*_0_ = 0.9 and *x*_0_ = 18.5. For the first initial guess, the number of iterations is set to *N* = 7, and it is *N* = 9 for the second initial guess. However, the absolute errors are smallest for the proposed method in both situations. Further, it may also be noted that the method given in Equation (2) failed for the convergence for both initial guesses, while the method given in Equation (1) diverges when the second initial guess is assumed.

**Problem 3 (fluid permeability in biogels [24]).**

The relation of the pressure gradient to the fluid velocity in porous medium (extracellular fiber matrix) can be defined with the specific hydraulic permeability via the following nonlinear model:

(40) $$\begin{array}{c} R_{f}x^{3}-20p{\left(1-x\right)}^{2}=0, \end{array}$$

where *R*_*f*_ stands for the radius of the fiber, *p* shows the specific hydraulic permeability, and *x* ∈ [0, 1] is the porosity of the medium. If we assume *R*_*f*_ = 100 × 10^−9^ and *p* = 0.4655, we obtain the following third-degree polynomial:

(41) $$\begin{array}{c} \zeta_{3}\left(x\right)=-100\times 10^{-9}x^{3}+9.3100x^{2}-18.6200x+9.3100. \end{array}$$

It is observed in Table 3 that the absolute error at the final iteration is smallest of all the errors and so is the absolute functional value while consuming reasonable amount of machine time computed in seconds. It is true in case of both initial guesses, that is, *x*_0_ = 1.5 and *x*_0_ = 2.5. For the first initial guess, the number of iterations is set to *N* = 9, and it is *N* = 10 for the second initial guess. However, the absolute errors are smallest in both situations.

**Problem 4 (law of population growth [26]).**

In the field of population dynamics, the following first-order linear ordinary differential equation is used:

(42) $$\begin{array}{c} P^{\prime }\left(t\right)=\kappa P\left(t\right)+v, \end{array}$$

where *P*(*t*) is the population at any time *t*, the constant birth rate of population is denoted by *κ*, and *v* shows the constant immigration rate. Solving the above linear differential model, we obtain its general solution as follows:

(43) $$\begin{array}{c} P\left(t\right)=P_{0}\exp\left(\kappa t\right)+\frac{v}{\kappa }\left(\exp\left(\kappa t\right)-1\right), \end{array}$$

where *P*_0_ is the initial population. Using the initial condition and values of the other parameters given in [27], the birth rate can be determined with the help of following nonlinear equation:

(44) $$\begin{array}{c} \zeta_{4}\left(x\right)=1564-100\exp\left(x\right)-\frac{435}{x}\left(\exp\left(x\right)-1\right)=0, \end{array}$$

where *x* = *κ* is the required birth rate.

It is observed in Table 4 that the absolute error at the final iteration is smallest of all the errors and so is the absolute functional value while consuming reasonable amount of machine time computed in seconds for the approximate birth rate determined to be *κ* ≈ 1.01*e* − 01. It is true in case of both initial guesses, that is, *x*_0_ = 2.5 and *x*_0_ = 4.5. For the first initial guess, the number of iterations is set to *N* = 6, and it is *N* = 6 for the second initial guess. However, the absolute errors are smallest in both situations. Further, it may also be noted that the method given in Equation (1) failed for *x*_0_ = 2.5 and diverged for *x*_0_ = 4.5. Similarly, the methods given in Equations (2) and (6) diverged for *x*_0_ = 4.5.

**Problem 5 (neurophysiology application [28, 29]).**

The nonlinear model consists of the following six equations:

(45) $$\begin{array}{c} x_{1}^{2}+x_{3}^{2}=1,\\ x_{2}^{2}+x_{4}^{2}=1,\\ x_{5}x_{3}^{3}++x_{6}x_{4}^{3}=c_{1},\\ x_{5}x_{1}^{3}+x_{6}x_{2}^{3}=c_{2},\\ x_{5}x_{1}x_{3}^{2}+x_{6}x_{4}^{2}x_{2}=c_{3},\\ x_{5}x_{1}^{2}x_{3}+x_{6}x_{2}^{2}x_{4}=c_{4}. \end{array}$$

The constants *c*_*i*_ in the above model can be randomly chosen. In our experiment, we considered *c*_*i*_ = 0, *i* = 1, ⋯, 4.

It is observed in Table 5 that the absolute error at the final iteration is smallest of all the errors for the proposed method given in (7) while consuming reasonable amount of machine time computed in seconds for the initial guess taken to be (*x*_10_, *x*_20_, *x*_30_, *x*_40_, *x*_50_, *x*_60_) = (1.8, 2.6, 1.5, 2.3, 3.8, 3.1). Further, it may also be noted that the methods given in Equations (4) and (5) diverged for this particular applied model. Thus, the proposed method (7) is highly accurate compared to other competitive methods.

## 7. Medical Science Models for Numerical Simulations

We have proposed a new three-step hybrid technique for dealing with nonlinear equations and real-world application problems in science and engineering. The proposed three-step hybrid technique has a convergence order of six and needs only five function evaluations. The newly proposed technique has a better efficiency index of 1.431. Using the Taylor series, the order of convergence and asymptotic error of the proposed three-step hybrid technique has been theoretically formulated in scalar and vector forms. Compared to other existing numerical techniques, the proposed three-step hybrid technique outperforms them in terms of absolute errors, absolute functional value computed during the last iteration, and machine time in seconds. Moreover, the proposed method has a minor absolute error, no matter the starting conditions are, for simulations of nonlinear models used in real-world medical science. The proposed technique's quick convergence is shown using polynomiography when applied to several complex-valued polynomials. Having said this, future research work would include implementing the proposed technique with memory while keeping time efficiency and computational complexity in mind and proving semilocal convergence. Regarding multiple solutions, the homotopy methods are useful. We will consider homotopy method while merging it with the existing approach to deal with the multiple roots. Such kinds of analyses will be carried out in future research studies.

## Figures and Tables

**Figure 1:** Flowchart of three-step sixth-order proposed method given in (7).

**Figure 2:** The polynomiographs simulated under the novel iterative technique for the complex-valued polynomials under consideration in Equation (37).

**Table 1:** Comparison of several methods with the proposed method under different initial guesses and different numbers of iterations for the blood rheology model given in (38).

Method	*ϵ* = |*x*_*N*_ − *x*_*e*_|	|*ζ*_1_(*x*_*N*_)|	Time	*ϵ* = |*x*_*N*_ − *x*_*e*_|	|*ζ*_1_(*x*_*N*_)|	Time
	*N* = 6, *x*_0_ = 2.0			*N* = 5, *x*_0_ = 4.2		
(1)	8.07e-07	1.15e-12	2.03e-01	1.04e-06	1.34e-10	1.71e-01
(2)	1.77e-77	6.63e-307	4.84e-01	Other sol.	—	—
(4)	4.02e-334	1.32e-2001	2.03e-01	1.16e-410	3.76e-2457	1.10e-01
(5)	Diverge	—	—	1.94e-411	8.30e-2462	3.91e-01
(6)	4.56e-138	5.43e-825	2.81e-01	2.72e-449	4.40e-2689	2.03e-01
(7)	1.08e-1166	4.93e-6997	2.34e-01	2.77e-675	7.15e-4045	1.40e-01

**Table 2:** Comparison of several methods with the proposed method under different initial guesses and different number of iterations for the blood flow model given in (39).

Method	*ϵ* = |*x*_*N*_ − *x*_*e*_|	|*ζ*_2_(*x*_*N*_)|	Time	*ϵ* = |*x*_*N*_ − *x*_*e*_|	|*ζ*_2_(*x*_*N*_)|	Time
	*N* = 7, *x*_0_ = 0.9			*N* = 9, *x*_0_ = 18.5		
(1)	5.72e-03	6.05e-01	1.56e-01	Diverge	—	—
(2)	Failed	—	—	Failed	—	—
(4)	5.62e-245	1.78e-1454	2.66e-01	2.27e-345	7.64e-2057	1.88e-01
(5)	7.77e-245	1.25e-1453	2.82e-01	3.61e-345	1.26e-2055	3.75e-01
(6)	1.65e-277	1.12e-1649	1.56e-01	1.23e-210	1.93e-1248	2.50e-01
(7)	2.05e-574	4.16e-3431	1.50e-01	3.08e-1013	4.81e-6064	2.18e-01

**Table 3:** Comparison of several methods with the proposed method under different initial guesses and different number of iterations for the blood flow model given in (39).

Method	*ϵ* = |*x*_*N*_ − *x*_*e*_|	|*ζ*_3_(*x*_*N*_)|	Time	*ϵ* = |*x*_*N*_ − *x*_*e*_|	|*ζ*_3_(*x*_*N*_)|	Time
	*N* = 9, *x*_0_ = 1.5			*N* = 10, *x*_0_ = 2.5		
(1)	9.75e-04	8.85e-06	2.81e-01	1.46e-03	1.99e-05	2.50e-01
(2)	2.07e-04	3.24e-08	7.34e-01	5.85e-02	1.43e-02	1.20e+00
(4)	1.34e-160	5.87e-944	2.18e-01	1.73e-293	2.71e-1741	2.81e-01
(5)	2.38e-74	9.44e-424	3.28e-01	1.43e-09	4.43e-35	4.22e-01
(6)	1.18e-170	2.67e-1004	4.21e-01	8.72e-381	4.45e-2265	2.97e-01
(7)	5.89e-628	4.23e-3748	3.03e-01	1.26e-1082	4.07e-6476	2.61e-01

**Table 4:** Comparison of several methods with the same number of iteration.

Method	*ϵ* = |*x*_*N*_ − *x*_*e*_|	|*ζ*_4_(*x*_*N*_)|	Time	*ϵ* = |*x*_*N*_ − *x*_*e*_|	|*ζ*_4_(*x*_*N*_)|	Time
	*N* = 6, *x*_0_ = 2.5			*N* = 6, *x*_0_ = 4.5		
(1)	1.01e-04	6.50e-06	3.12e-01	Diverge	—	—
(2)	Failed	—	—	Failed	—	—
(4)	2.34e-841	1.03e-5042	3.44e-01	5.00e-184	9.77e-1099	4.22e-01
(5)	2.97e-841	4.27e-5042	4.69e-01	5.27e-184	1.34e-1098	5.62e-01
(6)	4.53e-1088	3.25e-6524	4.22e-01	Failed	—	—
(7)	4.04e-1176	2.71e-7051	3.44e-01	3.70e-347	1.59e-2077	3.90e-01

**Table 5:** Comparison of several methods with the same number of iterations (*N* = 5) while the initial guess is set to be (*x*_10_, *x*_20_, *x*_30_, *x*_40_, *x*_50_, *x*_60_) = (1.8, 2.6, 1.5, 2.3, 3.8, 3.1).

Method	**ϵ**_*N*_ = |**x**_*N*_ − **x**_*e*_|	Time
(1)	2.26e-60	6.30e-02
(4)	3.08e-2000	1.88e-01
(5)	Diverge	—
(6)	Diverge	—
(7)	2.63e-2474	1.72e-01

## Data Availability

No data is used during the study.
